The article "Relationship between PLR and Clinicopathological Characteristics of Patients with Advanced NSCLC and Its Predictive Value for the Efficacy of Chemotherapy and Prognosis" was retracted in 2023. Reasons: signs of a paper mill; suspected computer-generated content; unreliable results or conclusions; concerns about the data.

# Relationship between PLR and Clinicopathological Characteristics of Patients with Advanced NSCLC and Its Predictive Value for the Efficacy of Chemotherapy and Prognosis

**DOI:** 10.1155/2022/5811219

**Published:** 2022-09-30

**Authors:** Jianming Zhao, Yiping Pan, Yu Sheng, Jun Sun

**Affiliations:** Department of Thoracic Surgery, Jinhua Guangfu Hospital, Jinhua, Zhejiang 321001, China

## Abstract

**Objective:**

To investigate the relationship between blood platelet-to-lymphocyte ratio (PLR) and clinicopathological characteristics of patients with advanced non-small cell lung cancer (NSCLC) and evaluate the value of PLR for predicting the efficacy of chemotherapy and prognosis.

**Methods:**

The clinical data of 175 patients with advanced NSCLC diagnosed from March 2017 to December 2018 in our hospital were retrospectively analyzed, and the data of 175 healthy subjects from our hospital physical examinations were included. The platelet was detected by using a blood cell analyzer to calculate PLR. According to the average PLR value (197) before chemotherapy, 175 patients were divided into the low PLR group (=78) and the high PLR group (=97). The relationship between the expression levels of PLR and clinicopathologic features was analyzed, and the Kaplan–Meier survival curve was used to analyze the relationship between the expression levels of PLR and prognosis.

**Results:**

The results showed that prechemotherapy PLR levels were significantly higher in NSCLC compared with the healthy subjects (*P* < 0.05). After 4 cycles of chemotherapy, the PLR levels were significantly lower than those during prechemotherapy (*P* < 0.05). The proportion of TNM (IV) stage cases in the low PLR group was lower than that in the high PLR group (*P* < 0.05). The total effective rate of the first-line chemotherapy was 46.9% (82/175). The effective rate of IIIb staging was higher than that in IV staging (*P* < 0.05), and the effective rate of the low PLR group was higher than that in the high PLR group (*P* < 0.05). Multivariate logistic analysis showed that TNM stage 4 and high PLR level were the independent risk factors for the efficacy of the first-line chemotherapy in patients with advanced NSCLC (*P* < 0.05), and the high PLR level was an independent risk factor affecting the prognosis of patients with advanced NSCLC. The median overall survival (OS) of patients with the low PLR group was 20.8 months, higher than the 12.0 months of patients with the high PLR group (*P* < 0.05).

**Conclusion:**

PLR might have a certain clinical significance for predicting the TNM staging of NSCLC and can provide important diagnostic and prognostic results for patients.

## 1. Introduction

Lung cancer is one of the most common malignant tumors worldwide, with the highest morbidity and mortality. Non-small cell lung cancer (NSCLC) is the main type of lung cancer, accounting for about 80%–85% of lung cancers. 70% of NSCLC patients have reached an advanced stage when they are found, with a high degree of malignancy and a short survival time. The 5-year survival rate of patients with stage IIIb NSCLC is only 26% [1–3]. Chemotherapy is currently one of the main treatments for advanced NSCLC, which can effectively prolong the survival time of patients, although there are still many defects. However, there is currently a lack of indicators with a relatively low cost and high specificity to effectively reflect the severity of NSCLC and evaluate the efficacy of chemotherapy. The levels of inflammatory factors play an irreplaceable role in the evaluation of the development and prognosis of tumors; among them, the peripheral blood platelet-lymphocyte ratio (PLR) is an easily obtained inflammatory index, and the combination of platelets and lymphocytes, which can better reflect the systemic inflammatory state [4, 5]. In addition, PLR is also closely related to the staging of solid tumors, chemotherapy, and surgical prognosis [6, 7]. In this study, the clinical data of 175 patients with advanced NSCLC were collected, and a retrospective cohort analysis was performed to explore the relationship between peripheral blood PLR levels and their clinicopathological characteristics in patients with advanced NSCLC and to evaluate the predictive value of PLR for the chemotherapy efficacy.

The article "Relationship between PLR and Clinicopathological Characteristics of Patients with Advanced NSCLC and Its Predictive Value for the Efficacy of Chemotherapy and Prognosis" was retracted in 2023. Reasons: signs of a paper mill; suspected computer-generated content; unreliable results or conclusions; concerns about the data.

## 2. Materials and Methods

### 2.1. Clinical Data

The clinical data of 175 patients with advanced NSCLC who were diagnosed and treated in our hospital from March 2017 to December 2018 were retrospectively collected, including gender, age, smoking history, pathological type, TNM stage, and performance status (PS). There were 115 males and 60 females, ranging in age from 32 to 78 years old, with an average age of (68.72 ± 8.53) years old. There were 98 cases with a smoking history and 77 cases without a smoking history. There were 94 cases of squamous cell carcinoma, 71 cases of adenocarcinoma, and 10 cases of large cell carcinoma. TNM staging lists 106 cases of stage IIIb and 69 cases of stage IV. PS score: 0–1 points in 123 cases (patient's physical function of was completely normal or he had only mild symptoms); ≥2 points in 52 cases (patients with tumor-related symptoms need to stay in bed for part of the day, or even worse). Inclusion criteria are as follows: (1) patients met the diagnostic criteria for NSCLC and were confirmed by pathological diagnosis [8]; (2) the TNM stage is stage IIIb (T4, N2, and M0 or T1a-4, N3, and M0) or stage IV (any of *T*, any of *N,* and M1a-1b) [9]; (3) the patient's estimated survival was greater than 3 months; (4) no acute infection within 2 weeks before admission; and (5) complete case data and follow-up data. Exclusion criteria are as follows: (1) patients with severe heart, lung, liver, or kidney insufficiency; (2) patients with other malignant tumors. At the same time, 175 healthy volunteers who underwent physical examination were included in our hospital, including 112 males and 63 females, aged 30–76 years, with an average age of (67.84 ± 8.48) years. There was no significant difference in general data such as gender and age between the two groups (*P* < 0.05); the two groups were comparable.

The article "Relationship between PLR and Clinicopathological Characteristics of Patients with Advanced NSCLC and Its Predictive Value for the Efficacy of Chemotherapy and Prognosis" was retracted in 2023. Reasons: signs of a paper mill; suspected computer-generated content; unreliable results or conclusions; concerns about the data.

### 2.2. Research Methods

#### 2.2.1. Evaluation of Curative Effect

All patients received chemotherapy, 21 days as a cycle, and at least 4 cycles of treatment. According to the evaluation criteria of efficacy [10], efficacy is divided into complete remission (CR), partial remission (PR), stable disease (SD), and progressive disease (PD). All patients were evaluated for short-term efficacy after four cycles of treatment. The effective rate = (CR cases + PR cases)/total cases × 100%.

#### 2.2.2. Blood Sample Collection and Testing

5 ml of fasting peripheral venous blood was collected from patients with NSCLC before and after chemotherapy and healthy volunteers. The blood cytology test was performed with an automatic blood routine analyzer. Reference range: platelet (PLT) count is (100–300) × 10^9^/L, lymphocyte (LY) count is (1.1–3.2) × 10^9^/L, and PLR is calculated. The range of PLR was 138.9–288.6, and the mean PLR (197) was taken as the cut-off value. Patients were divided into the low PLR group (*n* = 78) and the high PLR group (*n* = 97) according to the level of PLR.

#### 2.2.3. Follow-up

All patients were followed up regularly by outpatient or telephone after discharge, and the deadline for follow-up was December 31, 2019. Overall survival (OS) time refers to the time from the date of receiving chemotherapy to the time of death or last follow-up.

### 2.3. Statistical Processing

SPSS 22.0 software was used for processing, measurement data were expressed as the mean ± standard deviation ($\bar{x}$ ± *s*), comparison between groups was expressed by a *t*-test, enumeration data were expressed by (%), and comparison between groups was expressed by the *χ*^*2*^ test. The effective rate and OS time factors affecting it were analyzed by using a logistic regression model. Survival analysis was performed by the Kaplan–Meier method, the OS curve was drawn, and the comparison was performed by the log-rank test. *P* < 0.05 means the difference is statistically significant.

The article "Relationship between PLR and Clinicopathological Characteristics of Patients with Advanced NSCLC and Its Predictive Value for the Efficacy of Chemotherapy and Prognosis" was retracted in 2023. Reasons: signs of a paper mill; suspected computer-generated content; unreliable results or conclusions; concerns about the data.

## 3. Results

### 3.1. Comparison of PLR Levels in Patients with Advanced NSCLC before and after Chemotherapy and in Healthy Volunteers

The level of PLR (197.38 ± 26.92) before chemotherapy in patients with advanced NSCLC was higher than that in healthy volunteers (132.09 ± 23.27), and the difference was statistically significant (*P* < 0.05). After 4 cycles of chemotherapy, the level of PLR (188.90 ± 29.22) in advanced NSCLC patients was lower than that (197.38 ± 26.92) before chemotherapy, and the difference was statistically significant (*P* < 0.05), as shown in Figure 1.

### 3.2. The Relationship between PLR Levels before Chemotherapy and Clinicopathological Characteristics in Patients with Advanced NSCLC

There was no significant difference between the PLR level before chemotherapy and gender, age, smoking status, PS score, and pathological type in advanced NSCLC patients (*P* < 0.05). However, the proportion of TNM (IV) stage cases in the low PLR group was lower than that in the high PLR group; the differences were statistically significant (*P* < 0.05), as shown in Table 1.

### 3.3. Comparison of Effective Rate and OS Time in Patients with Advanced NSCLC

The effective rate of first-line chemotherapy in advanced NSCLC patients was 46.9% (82/175), and there was no significant difference with gender, age, smoking status, PS score, or pathological type (*P* < 0.05), and the effective rate in the stage IIIb group was higher than that in the stage IV group; the effective rate of the low PLR group was higher than that of the high PLR group, and the difference was statistically significant (*P* < 0.05). There was no significant difference between the median OS time and gender, age, smoking status, PS score, pathological type, and TNM staging of patients (*P* < 0.05). The median OS time in the low PLR group was higher than that in the high PLR group, and the difference was statistically significant (*P* < 0.05), as shown in Table 2.

### 3.4. Multivariate Logistic Analysis on Factors Affecting Efficacy of Chemotherapy and OS Time in Patients with Advanced NSCLC

Multivariate logistic analysis showed that TNM stage 4 and a high PLR level were the independent risk factors for the efficacy of first-line chemotherapy in patients with advanced NSCLC (*P* < 0.05), as shown in Table 3. The high PLR level was an independent risk factor affecting the prognosis of patients with advanced NSCLC (*P* < 0.05), as shown in Table 4.

### 3.5. The Relationship between Different PLR Levels and Prognosis of Patients

As of December 31, 2019, all 175 cases were followed up, of which 45 died. The median OS time of patients in the low PLR group was 20.8 months, which was higher than the median OS time of 12.0 months in the high PLR group, *P*=0.020 by the log-rank test, as shown in Table 2 and Figure 2.

The article "Relationship between PLR and Clinicopathological Characteristics of Patients with Advanced NSCLC and Its Predictive Value for the Efficacy of Chemotherapy and Prognosis" was retracted in 2023. Reasons: signs of a paper mill; suspected computer-generated content; unreliable results or conclusions; concerns about the data.

## 4. Discussion

The incidence and mortality of lung cancer are high all over the world, especially in China. In addition, NSCLC is the most common type of lung cancer, and it is difficult to find it in the early stages. At present, the commonly used treatment of NSCLC in clinical practice is mainly chemotherapy. However, there is still a lack of specific evaluation indicators for evaluating the severity of NSCLC and the efficacy of chemotherapy [11–13]. In recent years, PLR, as a biochemical indicator with strong operability, stable results, and low cost, has been favored by researchers. Current studies [14, 15] have shown that PLR has good predictive value in the evaluation and prognosis of solid tumors such as gastrointestinal tumors. However, there are few reports on the use of PLR to evaluate the efficacy of chemotherapy in advanced NSCLC. Therefore, this study retrospectively evaluated the relationship between PLR levels and their clinicopathological characteristics and the predictive value of PLR for the efficacy of chemotherapy in patients with advanced NSCLC.

The results of this study showed that the PLR of patients with advanced NSCLC before chemotherapy was higher than that of healthy volunteers. After receiving 4 cycles of chemotherapy, PLR in patients with advanced NSCLC was lower than before chemotherapy. When activated PLT is combined with tumor cells, PLT can prevent tumor cells from being detected and attacked by human immune cells and produce vascular endothelial growth factor and transforming growth factor beta to promote the growth of tumor cells. In addition, PLT can also produce a variety of cytokines, such as interleukin IL-1*β*, IL-6, and IL-12, which in turn promote the production of PLT by megakaryocytes and inhibit the secretion of LY, leading to an increase in PLR in patients. [16–18]. During the course of chemotherapy, the tumor cells in the patient's body were continuously killed, the inflammatory response decreased, the immune response increased, the secretion level of PLT decreased, and the secretion level of LY increased, which led the patients' PLR decreasing after chemotherapy. This may suggest that the changes of PLR in the peripheral blood of NSCLC patients can reflect the degree of disease and the number of tumor cells in the body to a certain extent.

The results of this study showed that the PLR level of patients was closely related to TNM staging, and the higher the TNM staging was, the higher the PLR level was. This suggests that the level of PLR is closely related to the disease progression and pathological development of NSCLC, which provides good evidence for PLR as a relatively common indicator for early screening of NSCLC.

The article "Relationship between PLR and Clinicopathological Characteristics of Patients with Advanced NSCLC and Its Predictive Value for the Efficacy of Chemotherapy and Prognosis" was retracted in 2023. Reasons: signs of a paper mill; suspected computer-generated content; unreliable results or conclusions; concerns about the data.

This study compared the effects of different clinicopathological features and PLR levels on the efficacy of chemotherapy and patients' OS time. The efficacy of chemotherapy was related to TNM staging and PLR. Among them, the effective rate of chemotherapy in stage IIIb patients was higher than that in stage IV patients, and the effective rate of chemotherapy in the low PLR group was higher than that in the high PLR group. The results of multivariate analysis showed that both TNM staging and PLR were independent influencing factors for the efficacy of chemotherapy. The survival time of the high PLR group was shorter than that of the low PLR group, and a high level of PLR is an independent risk factor affecting the prognosis of NSCLC patients. The results showed that a low PLR level represents better efficacy of chemotherapy and longer prognosis survival time to a certain extent, indicating that PLR has a good predictive value for the efficacy of chemotherapy and prognosis.

In conclusion, PLR has a certain significance in evaluating the TNM staging of advanced NSCLC patients and has important predictive value for the efficacy of chemotherapy and the prognosis evaluation of patients, which is worthy of clinical application. Due to the low cost and simple operation of PLR detection, it is recommended to use PLR as an inflammatory biochemical indicator for the prognosis of patients with advanced NSCLC, to help patients with advanced NSCLC choose a more individualized treatment plan in order to achieve better therapeutic efficacy and prolong survival time.

## Figures and Tables

**Figure 1:** Comparison of PLR levels in patients with advanced NSCLC before and after chemotherapy and in healthy volunteers. *Note.* Compared with healthy volunteers, ^*∗*^*P* < 0.05; compared with NSCLC patients before chemotherapy, ^#^*P* < 0.05.

**Figure 2:** Survival curves of patients with different PLR levels.

**Table 1:** Comparison of different clinicopathological features and PLR levels in patients with advanced NSCLC before chemotherapy (*n*, %).

Factor	Cases (*n* = 175)	Low PLR group (*n* = 78)	High PLR group (*n* = 97)	*χ* ^2^ value	*P* value
*Gender*					
Male	115	56 (48.7)	59 (51.3)	2.310	0.129
Female	60	22 (36.7)	38 (63.3)		

*Age (Years old)*					
<65	71	44 (56.4)	47 (48.5)	1.729	0.189
≥65	104	34 (43.6)	50 (51.5)		

*Smoking status*					
Yes	98	35 (44.9)	63 (64.9)	0.926	0.336
No	77	43 (55.1)	34 (35.1)		

*PS score (points)*					
0∼1	123	56 (45.5)	67 (54.5)	0.154	0.695
≥2	52	22 (42.3)	30 (57.7)		

*Pathological type*					
Squamous cell carcinoma	94	40 (42.6)	54 (57.4)	0.226	0.695
Adenocarcinoma	71	34 (47.9)	37 (52.1)		
Large cell carcinoma	10	4 (5.13)	6 (6.18)		

*TNM staging*					
IIIb	106	55 (51.9)	51 (48.1)	5.823	0.019
IV	69	23 (33.3)	46 (66.7)		

The article "Relationship between PLR and Clinicopathological Characteristics of Patients with Advanced NSCLC and Its Predictive Value for the Efficacy of Chemotherapy and Prognosis" was retracted in 2023. Reasons: signs of a paper mill; suspected computer-generated content; unreliable results or conclusions; concerns about the data.

**Table 2:** Comparison of effective rate and OS time in patients with advanced NSCLC (*n*, %).

Factor	Cases (*n* = 175)	Efficacy of chemotherapy	*χ* ^2^ value	*P* value	Median OS time (month)	*χ* ^2^ Value	*P* value
*Gender*							
Male	115	53 (46.1)	0.029	0.865	15.3	2.518	0.113
Female	60	29 (48.3)			14.9		

*Age (Years old)*							
<65	71	36 (50.7)	0.255	0.614	15.2	0.513	0.474
≥65	104	46 (44.2)			16.9		

*Smoking status*							
Yes	98	42 (42.9)	0.515	0.473	14.9	0.462	0.497
No	77	40 (43.5)			15.3		

*PS score (points)*							
0∼1	123	55 (44.7)	0.336	0.623	16.4	3.558	0.060
≥2	52	27 (51.9)			14.5		

*Pathological type*							
Squamous cell carcinoma	94	45 (47.9)	0.961	0.327	15.8	0.093	0.761
Adenocarcinoma	71	33 (44.0)			15.2		
Large cell carcinoma	10	4 (40.0)			15.0		

*TNM staging*							
IIIb	106	63 (59.4)	6.555	0.010	15.9	0.834	0.361
IV	69	19 (27.5)			14.8		

*PLR level*							
<197	78	48 (61.5)	6.937	0.037	20.8	3.393	0.047
≥197	97	34 (35.0)			12.0		

**Table 3:** Multivariate logistic analysis on the effect of chemotherapy in patients with advanced NSCLC (Assignment situation: “TNM stage IIIb” = “0”; “TNM stage IV = ”1”. “PLR < 197” = “0”; “PLR ≥ 197” = “1”).

Variable	*B* value	Walds	OR value	95% CI	*P* value
TNM staging	0.214	5.163	1.695	1.452∼1.894	0.042
PLR	0.089	4.734	1.306	1.069∼1.425	0.004

**Table 4:** Multivariate logistic analysis on affecting the prognosis of patients with advanced NSCLC (Assignment situation: “PLR < 197” = “0”; “PLR ≥ 197” = “1”).

Variable	*B* value	Walds	OR value	95% CI	*P* value
PLR	0.256	11.232	0.979	0.004∼1.712	0.001

## Data Availability

The data can be obtained from the author upon reasonable request.
